The article "The Association between Anthropometry Indices and Serum Concentrations of Gamma-Glutamyl Transferase, Alkaline Phosphatase, Alanine Aminotransferase, and Aspartate Aminotransferase" was published in 2021. Journal: Biomed Res Int.

# The Association between Anthropometry Indices and Serum Concentrations of Gamma-Glutamyl Transferase, Alkaline Phosphatase, Alanine Aminotransferase, and Aspartate Aminotransferase

**DOI:** 10.1155/2021/2365399

**Published:** 2021-11-22

**Authors:** Sahar Sobhani, Reihaneh Aryan, Mina AkbariRad, Elahe Ebrahimi Miandehi, Maryam Alinezhad-Namaghi, Seyyed Reza Sobhani, Sara Raji

**Affiliations:** ^1^Persian Cohort Research Center, Mashhad University of Medical Sciences, Mashhad, Iran; ^2^Clinical Research Development Unit, Imam Reza Hospital, Mashhad University of Medical Sciences, Mashhad, Iran; ^3^Department of Internal Medicine, Faculty of Medicine, Mashhad University of Medical Sciences, Mashhad, Iran; ^4^Department of Medical Informatics, School of Medicine, Mashhad University of Medical Sciences, Mashhad, Iran; ^5^Department of Nutrition, Faculty of Medicine, Mashhad University of Medical Sciences, Iran

## Abstract

**Background:**

Nowadays, metabolic syndrome (MetS) has become a great public health crisis that threatens too many lives worldwide. Many previous studies have been investigated the association between MetS and anthropometric indices. This study is aimed at investigating the association between anthropometric indices with gamma-glutamyl transferase (GGT), alkaline phosphatase (ALP), alanine aminotransferase (ALT), and aspartate aminotransferase (AST). We were using data from a large population-based cohort of seemingly healthy women and men.

**Methods:**

A total of 7216 participants were included in this study. The serum levels of GGT, ALP, ALT, and AST with bioimpedance measures were obtained at the time of enrollment. Multiple regression analysis was performed to assess the relationship between anthropometric indices and serum levels of the aforementioned laboratory tests.

**Results:**

Serum levels of GGT, ALP, ALT, and AST significantly correlated with body mass index (BMI). Only ALP had a significant association with visceral fat area (VFA). AST, ALT, and ALP levels had a positive correlation with 50 kHz whole-body phase.

**Conclusion:**

From the findings of this study, body mass index consistently appeared a good predictor of elevated hepatic enzymes and triglycerides. Thus, it can be helpful in clinical settings to identify patients at risk of nonalcoholic fatty liver disease, which is closely related to metabolic syndrome.

## 1. Introduction

Nowadays, metabolic syndrome (MetS) has become a great public health crisis that threatens too many lives worldwide [1]. This metabolic disorder occurs when at least three of the following medical conditions are being clustered: abdominal obesity, hypertriglyceridemia, low serum high-density lipoprotein (HDL) level, hyperglycemia, and hypertension [2]. Therefore, these conditions can potentially facilitate type 2 diabetes mellitus, chronic kidney disease, and cardiovascular disease and finally lead to increased mortality risk [3]. Many previous studies have investigated the association between MetS and anthropometric indices, but the best anthropometric indicator is not known to predict MetS incidence [4]. However, extensive epidemiological studies on the Iranian, Chinese, and Qatari adult populations demonstrated that waist circumference (WC) was highly associated with the MetS as its best indicator, while waist-to-height ratio (WHtR) was considered the best anthropometric index for MetS prediction in Japanese and Italian adults [5, 6].

The article "The Association between Anthropometry Indices and Serum Concentrations of Gamma-Glutamyl Transferase, Alkaline Phosphatase, Alanine Aminotransferase, and Aspartate Aminotransferase" was published in 2021. Journal: Biomed Res Int.

The fact that the liver is known as the vital organ in metabolic regulation is not a secret [7]. According to recent studies, liver function tests (LFTs), including serum concentration of aspartate transaminase (AST), alanine transaminase (ALT), alkaline phosphatase (ALP), and gamma-glutamyl transferase (GGT), can be valuable parameters in evaluating one's metabolic status, especially investigating cardio-metabolic disorders [8]. Interestingly, several studies have indicated a strong direct association between LFTs and MetS [9, 10]. Having attention to the liver metabolic pathways demonstrates that this multifunctional organ has a prominent role in regulating serum lipid profiles such as HDL, low-density lipoprotein (LDL), and triglyceride [11]. Obviously, each of these fatty components can eventually make the MetS incidence more probable [12]. Therefore, LFTs and liver enzymes can be associated with the state of lipid metabolism and play a role in metabolic disorders, including MetS [13, 14].

According to what was stated, it can be deduced that anthropometric indices, liver function, and metabolic status would be related to each other; in a detailed view, we hypothesized that anthropometric indices could be associated with the serum concentration of GGT, ALP, and liver enzymes and as key components of the metabolic disorders and MetS. Therefore, we investigated this hypothesis in a large population in Iran to demonstrate whether this association is established or not.

## 2. Material and Method

### 2.1. Setting and Participants

The PERSIAN Organizational Cohort Study in Mashhad (POCM) is a study of lifestyle and risk factors for noncommunicable diseases. Details of POCM have been reported previously [15]. This study was planned to recruit 12,000 employees (aged 30-70 years) in Mashhad, northeast of Iran. The detailed national protocol has been published elsewhere [16]. Baseline assessments were obtained by face-to-face interviews or examinations. The questionnaires consist of demographic characteristics, physical activity, personal and familial medical history, medication profile, and smoking, and alcohol use was collected by a standardized questionnaire [16]. Basic consent was obtained from all participants before entering the study. The study protocol was in accordance with the principles laid down in the Helsinki declaration and has been approved by the national and regional ethics committee (IR.MUMS.REC.1395.526; January 2017).

The article "The Association between Anthropometry Indices and Serum Concentrations of Gamma-Glutamyl Transferase, Alkaline Phosphatase, Alanine Aminotransferase, and Aspartate Aminotransferase" was published in 2021. Journal: Biomed Res Int.

### 2.2. Study Measurements and Clinical Assessments

*Bioimpedance and anthropometric measurements*: the bioimpedance test was performed using the InBody 770 body analyzer (InBody Corporation, Seoul, South Korea). The participations were asked to abstain from caffeine consumption for at least 24 hours and drinks and foods for at least four hours prior to the test. The participants were required to stand motionless, keeping the standard position (standing barefoot on the footplates while holding hand electrodes with straight arms and no touches in the armpits area). The height and body circumferences (waist and hip) were measured to the nearest one decimal point in centimeters, while the participant was shoeless and had light underclothes. The pregnant women and the patients who had implanted pacemakers were excluded from the body analysis.

#### 2.2.1. Laboratory Measures

All of the laboratories finding, such as liver enzymes, FBS, TG, LDL, HDL, and total cholesterol in POCM, were measured after 10-12 hours fasting in the morning (BT1500 auto analyzer, Biotechnical Instruments, Rome, Italy).

### 2.3. Statistical Analysis

Baseline characteristics of the study population were dichotomized based on men and women. Continuous variables were expressed as mean ± standard deviation, and discrete variables were expressed as percentages. Comparisons of categorical variables were performed by chi-square test, and analyses of continuous variables were performed by independent-samples *T*-test and Mann–Whitney. Multivariate linear regression analysis was used to determine the relationship between biochemical factors as dependent variables and measures of sex, age, WHR, BMI, TBW, VFA, and 50 kHz whole-body phase angle and measure circumferences of hip, BFM, TG, LDL, and HDL as independent variables. All analyses were performed using SPSS software version 22.

## 3. Results

A total of 7216 (3855 women and 3361 men) participants of the POCM from October 2017 to April 2021 were included in the present study. As shown Tables 1 and 2, men were older and had higher education level. Also, women had higher BMI, HDL, VFA, BFM, and measure circumference of chest and were less likely to be alcohol drinkers or smokers. Women and men had similar physical activity, but men had higher WC, whole-body phase angle, TBW, and FFM and higher GGT, ALT, AST, FBS, and LDL.

The article "The Association between Anthropometry Indices and Serum Concentrations of Gamma-Glutamyl Transferase, Alkaline Phosphatase, Alanine Aminotransferase, and Aspartate Aminotransferase" was published in 2021. Journal: Biomed Res Int.

As shown in Table 3, multivariate regression analysis using sex, age, WHR, BMI, TBW, VFA, LDL, HDL, TG, 50 kHz whole-body phase angle, and measure circumferences of hip and BFM as independent variables demonstrated that ALP levels were determined predominantly by sex, age, BMI, TG, LDL, and HDL but not with TBW and BFM (*P* > 0.05). The main determinants of GGT levels found were sex, age, BMI, LDL, HDL, and TG. ALT and AST levels had an inverse association with measure circumferences of hip (*β* − coefficient = −1.56, *P* = 0.001; *β* − coefficient = −1.05, *P* = 0.003).

AST, ALT, and ALP levels were a positive association with 50 kHz whole-body phase angle (*β* − coefficient = 0.15, *P* = 0.001; *β* − coefficient = 0.11, *P* = 0.004; *β* − coefficient = 0.17, *P* = 0.001), respectively, but GGT had no association with 50 kHz whole-body phase angle. AST, ALT, and GGT levels showed no significant relationship with VFA (*P* > 0.05). However, ALP had a significant association with VFA (*P* = 0.001). AST, ALT, ALP, and GGT levels had significantly positive correlations with TG, LDL, and HDL (*P* < 0.05) (Table 3).

## 4. Discussion

In our studied population of more than 7000 men and women, BMI was significantly correlated with ALT, AST, ALP, GGT, and TG.

Obesity has been a growing concern in recent years due to the close correlation between this condition and chronic diseases of lifestyle [17]. The worldwide prevalence of obesity nearly tripled between 1975 and 2016. The WHO adult BMI database in 2016 indicates that 39% of men and 40% of women were overweight, and about 11% of men and 15% of women were obese [18]. As shown in our study, obesity has also been identified as a significant contributing factor to increased serum levels of liver enzymes [19–21]. The “portal hypothesis” proposes this relationship is due to the high release of free fatty acids from the visceral fat depot into the portal circulation, leading to hepatic damage and nonalcoholic fatty liver disease (NAFLD) [22].

We found that only serum levels of ALP had a significant correlation with VFA, and the other laboratory test showed no significant correlation with this index. Ali AT et al. suggested that ALP is involved in controlling of intracellular lipid accumulation in human preadipocytes [23]. In a study on middle-aged Korean men regarding the association between serum ALP levels and development of the MetS over four years, ALP showed a significant association with abdominal obesity and risk of developing MetS [24].

The article "The Association between Anthropometry Indices and Serum Concentrations of Gamma-Glutamyl Transferase, Alkaline Phosphatase, Alanine Aminotransferase, and Aspartate Aminotransferase" was published in 2021. Journal: Biomed Res Int.

A study performed by Ghandehari et al. showed that waist circumference had the most accuracy in predicting liver injury in adults [25] which contrasts with our study as we found BMI to be a better consistent indicator for liver injury. This difference can be due to the difference in the method of diagnosing fatty liver in the two studies. In the previous study, a fibro scan was used, and the present study considered the toxic levels of liver enzymes. These variables may be associated with a low-grade fatty liver that has not yet increased liver enzymes.

Bioelectrical impedance analysis such as 50 kHz whole-body phase angle has been gaining attention because they are considered indexes of extra cellular (ECW) and intracellular water (ICW) distribution, body cell mass (BCM), and cellular integrity [26].

A Spanish study showed that low tertile of phase angle is a cardiovascular risk factor in obese patients [27]. Controversially, in our study, 50 kHz whole-body phase angle had a positive correlation with ALT, AST, ALP, and TG, as supported by a study done by Moreto et al. It can be deduced that 50 kHz whole-body angle is an indicator of good nutritional status in a healthy population and is not a good predictor of MetS [28].

ALP and GGT levels were positively correlated with age, while ALT was negatively correlated with age, and AST showed no such significance. A study performed by Dong et al. also showed that ALT levels, independent of metabolic syndrome components and other commonly used hepatic enzymes, decreased with age in both genders, while age did not affect AST levels [29]. The same results were reported in another study by Oliveira et al. in 2016 [30].

Sex differences in anthropometric indices seem to be inconsistent among different communities. In our studied population, women had higher BMI, HDL, WHR ratio, VFA, BFM, and chest circumference, while men had higher WC, LDL, TBW, FFM, neck circumference, and 50 kHz whole-body angle. In a study of 12,514 adults from Isfahan, Iran, women tended to have higher BMI, WHR, and also WC [31]. Controversially, in a study of 27,257 adults in China [32], men had significantly higher BMI.

Our male population had significantly higher serum levels of liver enzymes, TG, LDL cholesterol, and FBS along with lower serum levels of HDL cholesterol. These gender-based differences can be likely explained by gender disparities in gonad corticoids, body fat distribution, and lifestyle [33]. For instance, men were more likely to be smokers (*P* < 0.001) and drinkers (*P* < 0.001) in our study.

In this investigation, a large number of participants were included, and we implemented a population-based cohort design, which has never been done before on the population of Mashhad, the second largest city of Iran, regarding this subject. Although these findings may not translate to patients of other ethnicities, the results might still be widely applicable as they were mostly consistent with other studies around the world.

The article "The Association between Anthropometry Indices and Serum Concentrations of Gamma-Glutamyl Transferase, Alkaline Phosphatase, Alanine Aminotransferase, and Aspartate Aminotransferase" was published in 2021. Journal: Biomed Res Int.

Our study was not without limitations. We did not exclude risk factors other than obesity and central adiposity for liver diseases, such as taking certain medications, old blood transfusions, and family history of liver disease. The presence of participants with these risk factors, who may have had elevated liver enzymes for reasons above, may have affected the results.

## 5. Conclusion

From the findings of anthropometry indices, body mass index consistently appeared a good predictor of elevated hepatic enzymes and fatty liver disease. Other incidences such as waist circumference could not be a good predictor of fatty liver. Thus, it can be useful in clinical settings to identify patients at risk of nonalcoholic fatty liver disease, which is closely related to metabolic syndrome. BMI is an adequate and efficacious measuring tool to identify patients at risk of NAFLD and MetS. We recommend BMI as a screening tool to identify patients at high risk of MetS in Khorasan Razavi province.

## Figures and Tables

**Table 1:** Demographic characteristics of the participants.

Characteristics	Women (*n* = 3855)	Men (*n* = 3361)	*P* value
Age, years, mean (SD)	44.1 (9.2)	46.3 (8.3)	<0.001
Education, %			<0.001
Primary or below	3.2	1.8	
Middle school	21.6	14.1	
College or above	75.2	84.1	
Physical activity, %			0.958
Inactive	0.8	0.8	
Moderate	95.9	95.9	
Active	3.3	3.3	
Alcohol use, %			<0.001
Never	98.1	95.2	
Former	0.4	3.5	
Current	1.3	1.5	
Smoking, %			<0.001
Never	98.6	83.1	
Former	0.3	6.6	
Current	1.1	10.3	

**Table 2:** Biochemical and anthropometry parameters.

Characteristics	Women (*n* = 3855)	Men (*n* = 3361)	*P* value
Body mass index, kg/m^2^, mean (SD)	27.2 (4.2)	26.8 (5.1)	<0.001
Waist circumference, cm, mean (SD)	94.8 (10.7)	98.4 (8.9)	<0.001
Waist hip ratio, cm, mean (SD)	0.94 (0.067)	0.92 (0.054)	<0.001
Visceral fat area, cm, mean (SD)	137.8 (42)	102 (39)	<0.001
50 kHz whole-body phase angle, degree, mean (SD)	5.08 (0.5)	5.89 (0.6)	<0.001
Measure circumference of neck cm, mean (SD)	35.4 (3.1)	38.5 (2.4)	<0.001
Measure circumference of chest cm, mean (SD)	101.3 (6.8)	93.8 (6.9)	<0.001
Measure circumference of abdomen cm, mean (SD)	90.2 (10.1)	95.3 (11)	<0.001
Measure circumference of hip cm, mean (SD)	98.4 (3.7)	101.1 (6.2)	<0.001
Measure circumference of right arm cm, mean (SD)	31.9 (3.3)	33.5 (2.9)	<0.001
Measure circumference of left arm cm, mean (SD)	31.8 (3.2)	33.4 (2.9)	<0.001
Measure circumference of right thigh cm, mean (SD)	53.1 (4.1)	54.7 (4.3)	<0.001
Measure circumference of left thigh cm, mean (SD)	52.6 (3.9)	54.3 (4.1)	<0.001
Total body water, mean (SD)	29.9 (3.6)	42.7 (5.6)	<0.001
Body fat mass, mean (SD)	27.1 (7.8)	22.6 (7.7)	<0.001
Fat free mass, mean (SD)	40.7 (4.9)	57.2 (7.7)	<0.001
Triglycerides, mg/dl, mean (95% CI)	105.65 (55.40)	141.96 (80.18)	<0.001
GGT, U/L, mean (SD)	23 (20.06)	32.10 (21.35)	<0.001
AST, U/L, mean (SD)	20.21 (7.17)	23.98 (8.58)	<0.001
ALT, U/L, mean (SD)	20.90 (10.68)	30.55 (14.98)	<0.001
Fasting blood sugar, mg/dl, mean (SD)	94.62 (21.2)	102.53 (28.4)	<0.001
LDL cholesterol, mg/dl, mean (SD)	98.98 (30.524)	101.57 (31.59)	0.007
HDL cholesterol, mg/dl, mean (SD)	60.45 (13.40)	51.10 (10.62)	<0.001
Total cholesterol, mg/dl, mean (SD)	180.08 (36.9)	180.20 (36.8)	<0.001
ALP IU/L, mean (SD)	168 (59.8)	183 (51.5)	<0.001

The article "The Association between Anthropometry Indices and Serum Concentrations of Gamma-Glutamyl Transferase, Alkaline Phosphatase, Alanine Aminotransferase, and Aspartate Aminotransferase" was published in 2021. Journal: Biomed Res Int.

**Table 3:** Multiple regression analyses.

Model No.	Dependent variable	Independent variables	*β*-coefficient (*P*)	Adjusted *R*^2^ (*P*)
ALP		Sex	-0.31 (0.001)	0.08 (0.001)
		Age	0.06 (0.001)	
		WHR	0.12 (0.03)	
		BMI	-0.11 (0.02)	
		TBW	-0.02 (0.86)	
		VFA	0.61 (0.001)	
		50 kHz whole-body phase angle	0.16 (0.001)	
		Measure circumferences of hip	0.45 (0.27)	
		BFM	-0.09 (0.50)	
		HDL	0.03 (0.02)	
		LDL	0.07 (0.001)	
		TG	0.09 (0.001)	
GGT		Sex	-0.19 (0.001)	0.12 (0.001)
		Age	0.01 (0.001)	
		WHR	0.02 (0.95)	
		BMI	0.06 (0.04)	
		TBW	-0.30 (0.12)	
		VFA	0.14 (0.105)	
		50 kHz whole-body phase angle	-0.01 (0.48)	
		Measure circumferences of hip	-0.38 (0.32)	
		BFM	-0.13 (0.29)	
		TG	0.19 (0.001)	
		LDL	0.08 (0.001)	
		HDL	0.05 (0.001)	
AST		Sex	-0.18 (0.001)	0.12 (0.001)
		Age	0.01 (0.50)	
		WHR	-0.01 (0.82)	
		BMI	0.03 (0.03)	
		TBW	0.04 (0.66)	
		VFA	0.04 (0.62)	
		50 kHz whole-body phase angle	0.16 (0.02)	
		Measure circumferences of hip	-0.10 (0.02)	
		BFM	-0.12 (0.33)	
		TG	0.16 (0.001)	
		LDL	0.13 (0.001)	
		HDL	0.07 (0.001)	
ALT		Sex	-0.24 (0.001)	0.23 (0.001)
		Age	-0.05 (0.001)	
		WHR	-0.19 (0.3)	
		TBW	-0.23 (0.53)	
		VFA	-0.08 (0.30)	
		BMI	0.19 (0.004)	
		50 kHz whole-body phase angle	0.15 (0.001)	
		Measure circumferences of hip	-1.23 (0.001)	
		BFM	-0.56 (0.67)	
		TG	0.16 (0.001)	
		LDL	0.05 (0.001)	
		HDL	0.05 (0.001)	

Abbreviations: WHR: waist-hip ratio; BMI: body mass index; TBW: total body water; VFA: visceral fat area; BFM: body fat mass.

## Data Availability

The datasets used and/or analyzed during the current study are available from the corresponding author on reasonable request.
